The article "Combining Latent Factor Model for Dynamic Recommendations in Community Question Answering Forums" was retracted in 2023. Reasons: signs of a paper mill; compromised peer review; unreliable results or conclusions.

# Combining Latent Factor Model for Dynamic Recommendations in Community Question Answering Forums

**DOI:** 10.1155/2022/7191657

**Published:** 2022-06-24

**Authors:** Muhammad Usman, Farwa Ahmad, Usman Habib, Adeel Ashraf Cheema, Muhammad Umar Aftab, Muhammad Ahmad

**Affiliations:** ^1^Department of Computer Science, National University of Computer and Emerging Sciences, Islamabad, Chiniot-Faisalabad Campus, Chiniot 35400, Pakistan; ^2^Faculty of Computer Sciences and Engineering, GIK Institute of Engineering Sciences and Technology, Topi 23640, District Swabi, Khyber Pakhtunkhwa, Pakistan

## Abstract

Community Question Answering (CQA) web service provides a platform for people to share knowledge. Quora, Stack Overflow, and Yahoo! Answers are few sites where questioners post their queries and answerers respond to their respective queries. Due to the ease of use and quick responsiveness of the CQA platform, these sites are being widely adopted by the community. For better usability, there is a dire need to route the question toward the relevant answerers. To fulfil this gap, recommender systems play an important role in identifying the relevant answerers. To map the user interests more effectively, this research work proposed a dynamic feature representation of the latent user attributes for user profiling. The latent features are mapped by leveraging the Latent Dirichlet Allocation (LDA) for topic modelling of user data. The proposed recommendation model segments the user profile based on these latent user profiles incorporating the incremental learning of the users' interests to produce the relevant recommendations in near real time. The experimental setup generated recommendation lists of variable sizes and evaluated using multiple evaluation metrics, such as mean average precision, recall, throughput, and different quality metrics, such as discounted cumulative gain and mean reciprocal rank. The results showed that the proposed model provided a better quality of recommendations in CQA forums, which is promising for future research in this domain.

## 1. Introduction

In this digital era, more people are using the Internet for multi purposes, such as online business, community interactions, online gaming, and streaming content. People are exposed to problem when buying something online; that is, it not only requires enough information but also needs to make the right decisions with a huge pile of information. Nowadays, people always approach the Internet for searching for required products and services. With the Internet becoming the vital source of information, users rely on search to seek knowledge of the information. However, search engines do not suit the nonfactual questions, for example, which one is best local Chinese restaurant [1]. Similarly, Community Question Answering (CQA) web services provide a platform for users to post their questions to seek answers from other users. These services allow people to ask any question or to answer any question in a community of web service users. There are some sites where users can ask a question on any topic, whereas sites like Stack Overflow and Quora are more specified platforms. All these platforms are based on the control of human skills and the motivation of users to provide answers and share knowledge. Stack Overflow includes a rich graphical and user-friendly interface with so extensive features [2]. A summary of different community platforms is provided in Table 1.

The article "Combining Latent Factor Model for Dynamic Recommendations in Community Question Answering Forums" was retracted in 2023. Reasons: signs of a paper mill; compromised peer review; unreliable results or conclusions.

Recommender systems are proved to be effective at delivering the user an additional intelligent and practical data service by creating tangible product or service recommendations that are concerned with their learned preferences and requirements by combining the concepts of user identification, data filtering, and machine learning techniques [3]. Recommender systems are classified into three major categories based on the information filtering process. The content-based filtering (CBF) identifies the specific interests of items by analysing the descriptions or details of the item and provides recommendations for items based on similar items that a user has liked before [4, 5]. Collaborative filtering (CF) is the procedure of estimating or filtering the items by using the views or feedback of other users, and hybrid filtering combines filtering techniques to achieve better performance [6, 7].  Figure 1 shows the structure of hybrid recommender systems.

People are dependent on recommender systems intentionally or unintentionally to resolve the problem of information surplus [8, 9]. However, Recommender systems are proved to be the required solution for the problems of overwhelmed information on the Internet where it is very difficult for users to find the correct information at the right time as they provide better, dynamic, and customized information to the users [10, 11]. A major issue in CQA systems is to find the expert user to answer the question. This issue of recommending experts is also known as the expert finding or question routing problem [12, 13]. Experts are defined as the indefinite number of users who seem to provide answers of high quality to the questions posted based on the inputs discussed earlier [14]. Finding an expert for CQA is a challenging problem that appeared in many applications, like routing the questions and finding the best answers [15]. The recommendation system comprises the technologies that can aid in finding the appropriate experts for the users [16]. A naïve model representation is shown in Figure 2.

The article "Combining Latent Factor Model for Dynamic Recommendations in Community Question Answering Forums" was retracted in 2023. Reasons: signs of a paper mill; compromised peer review; unreliable results or conclusions.

However, CQA websites are dynamic where new users are joining; thus, interests of these users are changing with improved skills or expertise. Existing recommendation models can take ample amount of time and computation resources to retrain the model with the new data. These recommendation systems may need a lot of computations to deal with the updated information of new users. There is no such work designed to deal with the newly available information in best of our knowledge. So, there is a need to introduce a novel model that should be capable of generating dynamic recommendations about new information and could adapt the recommendation behaviour with the time efficiently.

In this paper, we propose a novel approach that deals with the information dynamically to recommend experts in the community question answering forums who can better satisfy the questions of users. The primary contributions of this paper are as follows:

- The proposed approach ensures that recommended experts can provide quality answers and updated recommendations are provided to the users without requiring a large amount of time for model training.
- This study proposes a novel mechanism to map the user data points with latent features projections. These latent projections are then aggregated to make user profiles.
- Proposed recommendation engine is based on the incremental clustering approach, which provides updated, efficient, and effective results based on incremental and updated information.
- Ranked recommendations are provided to users by analysing the latent features of the experts' profiles.

The organization of the paper is as follows: we discuss the related work followed by the methodology section and results. The results section is followed by a discussion section. Furthermore, the conclusion section is provided. At last, limitations and future works section is placed.

## 2. Related Work

Finding the expert in the CQA forums has been a challenging task so far as the real-time data generated by these sites is abundant and velocity is hyperactive. This abundance of data has posed a serious challenge to recommender systems to produce dynamic recommendations. Different research studies have been proposed in the literature to tackle the problem by leveraging many domains, such as machine learning, deep neural networks, and fuzzy inference systems. Huang et al. [17] have proposed a scheme for finding experts in multiple collaborative networks by using tree-guided tensor decomposition and matrix factorization to analyse user expertise. Yuan et al. [18] proposed a solution to find expert users in community question answering by focusing on the problem of low participation in these sites due to the unawareness of users about new questions. The authors of [19] considered the user's interest and expertise on the topics. They considered the problem of lack of work on user interests in previous research. Proposed study employed LDA and recommendations are generated by collaborative voting using user profiles.

The article "Combining Latent Factor Model for Dynamic Recommendations in Community Question Answering Forums" was retracted in 2023. Reasons: signs of a paper mill; compromised peer review; unreliable results or conclusions.

In [20], Ebesu et al. proposed an extension of supervised LDA through which collaborative effects in CQA sites are exploited and user profiles are modelled based on the topics in which they have expertise. Costa et al. [21] found that previous approaches consider the overall profiles or topics for finding experts. To provide a solution, they modelled the user expertise under tags rather than general topics or user profiles. They identified the expertise of users using the tags and voting scores of answerers in the community question answering sites. Kundu et al. [22] have proposed a method to find an expert in community question answering websites by estimating the ranking of user authority for every question. This proposed solution is based on the technique of performing analysis of links and similarities among topics between users and questions. The authors of [23] have proposed prediction approaches to predict who will answer a question. They performed prediction as soon as a question is created using limited information available. Proposed study applies feature-based prediction and social network-based predictions. The authors of [24] have proposed a method of finding expert based on the theme in query likelihood language (QLL). In this method, significance values are assigned to the words in the query that is based on their capabilities of representing a theme. Dataset from Yahoo! Answers is used for the evaluation of the proposed scheme.

Sahu et al. [25] considered the problem of lack of user evaluation in a specific domain. They identified if the user providing answers is authoritative in topics or not and applied statistical topic modelling to identify features. They used feature vector to acquire the classifier model for achieving identification of the topical authority of the answerer. The authors in [26] have analysed the answers of Stack Overflow with the questions to predict the best answer and perform analysis on the dataset to make it able to answer four research questions. The study proposed in [27] is the proposed algorithm that focuses on the elements of network structure and topic distribution of questions and answers. This algorithm is based on the structure of links between users and similarity of topics between users, questions, and answers. In this algorithm, topic distribution for users and questions is provided by LDA.

The article "Combining Latent Factor Model for Dynamic Recommendations in Community Question Answering Forums" was retracted in 2023. Reasons: signs of a paper mill; compromised peer review; unreliable results or conclusions.

Chi et al. [28] proposed a model for tag recommendation by using tags and their relative words. They empirically verify the relevance tag-content and proposed supervised topic model to generate the contented words by using either the normal tag-word or tag-relevance distribution. The authors of [29] proposed improved dynamic LDA to find domain experts by dividing the corpus according to time for dynamicity. To provide text topic mining of dynamic LDA, the authors determined the sets of text pieces in the overall time according to the features of text and considered the prior probability of the topic of text of the present time slice as the topic-word posterior probability distribution of the preceding time slice multiplied with its weight. Neshati et al. [12] have proposed two algorithms for predicting experts in future in community question answering forums. They have considered different features, like similarity of topics, development of topics, user behaviour, and topical transition, to predict the probability of a user becoming an expert in the future. Proposed algorithms are based on pointwise learning and pairwise learning [30] mechanisms. This work is like the Temporal Profile Based Model (TPBM) as both rely on the Markov assumption for modelling the change of a given user from a current topic to a future topic. Le and Shah [31] have predicted the possible answerers based on the content of questions and profiles of users. In the proposed scheme, the authors have utilized the past activities for generating the user's profile.

## 3. Proposed Methodology

This section describes the detailed method of our proposed approach. This model is divided into three modules (i.e., topic modelling, profile modelling, and recommendation engine).

### 3.1. Latent Dirichlet Allocation for Topic Modelling

Topic modelling is the class of approaches for text analysis that are used to analyse the groups of words together rather than to individually count these words for obtaining the dependency of the word's meaning on the wider perspective. This technique is used to extract underlying topics from a huge number of texts [32, 33]. There are several different approaches proposed for topic modelling, and among all these approaches, Latent Dirichlet Allocation (LDA) [34] is most popular in the field of data mining. Firstly, the topic modelling is applied to the user profiles to find the users' interests in certain topics. For this, we have implemented a Latent Dirichlet Allocation (LDA) scheme, which topicalizes a certain document. LDA provides us with users interested in certain topics.

The article "Combining Latent Factor Model for Dynamic Recommendations in Community Question Answering Forums" was retracted in 2023. Reasons: signs of a paper mill; compromised peer review; unreliable results or conclusions.

LDA observes all the words present in any of the given documents and provides identification of the topics to be present in that document [35]. It gives a generation of the topics, which is based on the occurrence of words from a given set of documents. In LDA, topics are probability distributions over the words [36]. LDA belongs to probabilistic generative model class, in which documents are represented as random combinations over latent topics that are characterized by the distribution of the words available in the document corpus. The algorithm used for LDA topic modelling made some assumptions about the vector dimensions of *z* known and fixed. Along with that, the word probabilities are parameterized by matrix *β* where *β*_*ij*_ = *p*(**w**^**j**^ = 1 | **z**^**i**^ = 1) is also fixed length that needs to be estimated along with the process. **N** is the ancillary variable that is independent of the generating variables (*θ* and *z*).

Dirichlet variable *θ* lies in the simplex if *θ*_*i*_ ≥ 0, ∑_*i*=1_^*k*^*θ*_*i*_=1 and has following probability density function:

(1) $$\begin{array}{c} \rho \left(\theta |\alpha \right)=\frac{\Gamma \left(\sum_{i=1}^{k}\alpha_{i}\right)}{\prod_{i=1}^{k}\Gamma \left(\alpha_{i}\right)}\theta_{1}^{\alpha_{i}-1}\ldots \theta_{k}^{\alpha_{k}-1}, \end{array}$$

where *α* is the *k*-vector with *α*_*i*_ > 0 and Γ(*x*) is the gamma function. Given the parameters *α* and *β*, the joint distribution of the topic mixture *θ* can be calculated as in the following equation for a given set of *N* topics *z* and set of *N* words **w**.

(2) $$\begin{array}{c} \rho \left(\theta ,z,w|\alpha ,\beta \right)=\rho \left(\theta |\alpha \right)\prod_{n=1}^{N}\rho \left(z_{n}|\theta \right)\rho \left(w_{n}|\beta \right), \end{array}$$

(3) $$\begin{array}{c} \rho \left(w|\alpha ,\beta \right)=\int \rho \left(\theta |\alpha \right)\left(\prod_{n=1}^{N_{\text{d}}}\sum_{z_{n}}\rho \left(z_{\text{d}n}|\theta \right)\rho \left(w_{n}|z_{n},\beta \right)\right)\text{d}\theta . \end{array}$$

Equation (3) represents the marginal distribution of a document. The corpus probability can be calculated by taking a product of marginal probabilities of single document as shown in the following equation.

(4) $$\begin{array}{c} \rho \left(\text{D}|\alpha ,\beta \right)=\prod_{\text{d}=1}^{M}\int \rho \left(\theta_{\text{d}}|\alpha \right)\left(\prod_{n=1}^{N_{\text{d}}}\sum_{z{\text{d}}_{n}}\rho \left(z_{\text{d}n}|\theta_{\text{d}}\right)\rho \left(w{\text{d}}_{n}|z_{\text{d}n},\beta \right)\right)\text{d}\theta_{\text{d}}. \end{array}$$

In our approach, all the answers provided by a user are considered as a document and the set of all the documents are given as input to the LDA model, which gives the topics to that document. In this way, can get the users interesting topics as shown in Algorithm 1.

The article "Combining Latent Factor Model for Dynamic Recommendations in Community Question Answering Forums" was retracted in 2023. Reasons: signs of a paper mill; compromised peer review; unreliable results or conclusions.

### 3.2. Feature Sampling for Latent Profiles

In recommender systems, the projection of user and item in latent factor space is important. These projections can solve the problems of diverse and dynamic recommendations as per the users' interests. This idea is leveraged in this paper to represent each user in the recommendation engine in its latent space. However, to make the latent trajectories more effective, a weight must be given only to important factors that may affect the overall quality of the recommendations. For this purpose, this study uses the popular term frequency to evaluate the importance of the words so that only important feature words go as input to the LDA [36]. Term frequency (*tf*) shows how many times a word occurs in the document in a corpus. It can be called the fraction of the frequency of the word in a document to the total number of words that appeared in the document. The value of *tf* increases by increasing the number of occurrences of the word in the document.

(5) $$\begin{array}{c} tf_{ij}=\frac{n_{i},j}{\sum_{k}n_{i,j}}. \end{array}$$

Inverse document frequency (IDF) is the measure of the common or rare words in the document. A high value of IDF means the word is rare in the document; it can be calculated as IDF = log(*N*/*df*_*i*_). Finally, the *tf*-*idf* is simply taken as the product of *tf* and *idf* as shown below:

(6) $$\begin{array}{c} tf-i\text{d}f,=tf_{i}*\;i\text{d}f_{i}. \end{array}$$

Here, *tf*_*i*_ is the number of existing terms in the document *j* and *idf*_*i*_ is the number of documents containing a term *i*.

### 3.3. Profile Segmentation Modelling

The second module of our approach is profile modelling. In this module, the topics generated from LDA topic modelling is clustered by using *k*-means clustering and the user profile is generated using the cosine similarity between the topic and the user. Elbow method is used in determining the number of clusters to be generated in our model.

*K*-means is considered as one of the most well-known partitioning algorithms as it is based on deciding the starting number of clusters and defining the initial value of centroid [37, 38]. This algorithm needs precise numbers for deciding the clusters numbers; unstable grouping of data can occur because of the variation in the initial center of the cluster. Algorithm 2 explains the algorithm for *K*-means clustering. This algorithm is a distance-based partitioning algorithm that partitions the data into a clusters number in numerical form [39, 40]. Therefore, the output of the *K*-means algorithm is dependent on the value of the cluster center selected.

The article "Combining Latent Factor Model for Dynamic Recommendations in Community Question Answering Forums" was retracted in 2023. Reasons: signs of a paper mill; compromised peer review; unreliable results or conclusions.

*K*-means clustering is used to segment the similar topics into cluster for each user. These obtained topics are provided to the *K*-means clustering algorithm as input and it clusters the given topics based on Euclidean distance used to find the closeness of the given data points. These generated clusters show how close a topic is to another. Closely related topics are partitioned into a cluster. Clusters are generated according to the algorithm explained above. However, there are many approaches that can be used to generate clusters, but the scope of the proposed user modelling is not overlapping clusters right now. Although the *K*-means algorithm for clustering is a famous and simple clustering method, there exists a problem in the identification of the number of clusters to be generated. The elbow method is a fundamental process to define the accurate value for the number of clusters to be formed [41]. This method helps in the selection of an optimal number of clusters by fitting the model with a values range for *K*. We used elbow method for determining the optimized or the suitable number of clusters.

Elbow method considers the variants percentage as the function of the number of clusters. Based on the concept that there must be the existence of an optimal number of *K*-means clusters, having extra clusters does not supplement the model substantially [42]. In the process, it adds the value of *k* for each cluster number and calculates the Sum Square Error (SSE) by the following equation.

(7) $$\begin{array}{c} \text{SSE}=\sum_{k=1}^{k}\sum_{x_{i}s_{k}}{\left(x_{i}-c_{k}\right)}^{2}. \end{array}$$

SSE can be defined as the sum of the average Euclidian distance at every point across the centroid [43]. In the above equation, *S*_*k*_ is the cluster *k*, *x*_*i*_ is the point of sample in *S*_*k*_, and *C*_*k*_ is the mean of all samples in *S*_*k*_. SSE is the error of clustering in all the samples representing the good or bad result of sampling. The value of SSE is reduced progressively with the increase of value of *K*, whereas the value of *k* is reduced significantly when the value of *k* is smaller than actual clusters numbers. The rate of convergence return on the value of *K* is reduced rapidly as *k* becomes equal to the actual number of clusters. This means that the drop rate of SSE fell dramatically and starts fading. The SSE is useful for the selection of the appropriate number of clusters by fitting the model on a different range of values for *K*. For each value of *K*, the error between the centroid is observed and displayed in Figure 3. It can be noted from Figure 3 that there has been a visualization effect of “arm” in the behaviour of error and number of clusters. The error is exponentially decreasing as the value of *K* is increased. We fitted the *K*-means model for different value ranges of *K*, as shown in the diagram, and our model displayed an “elbow” effect at value range from 35 to 40. The elbow effect indicates that underlying model fits good at *K*-value at 38.

The article "Combining Latent Factor Model for Dynamic Recommendations in Community Question Answering Forums" was retracted in 2023. Reasons: signs of a paper mill; compromised peer review; unreliable results or conclusions.

### 3.4. Incremental Learning

As the CQA sites are dynamic, there is a continuous increase in the information. New users are adding continuously; content is updating day by day; there is a need for such a model, which can deal with such a huge information update and provide the results based on the new and updated information effectively. In this model, we propose an incremental clustering approach [44], which deals with the new information without taking time required for retraining the models on every update. In the process of incremental *k*-means clustering [44], clustering is applied to the collected data blocks. *K*-means algorithm is performed on each data block and the final centers generated on the previous block are used as the initial centers for the next block. The algorithm for incremental clustering is explained in Algorithm 3.

When a new data point has arrived, incremental clustering calculates its distance with each cluster and then it will move to the cluster to which it is much close based on the measured distance. Groups of the new data available in the database are made into blocks and *k*-means clustering approach is applied on each block one by one. The centroids calculated after applying *k*-means clustering on one block are then used as the initial center points for the block to be clustered using *k*-means approach. This makes our model more efficient than other proposed models.

### 3.5. Recommendation Model

This module consists of two main steps for providing recommendations. The first step is to find similarities between the topics of questions posted and the candidate users by using the cosine similarity. The second step consists of the recommendation rank, which is based on three main features (i.e., reputation of the user, score, and accepted number of answers). Cosine similarity is used in text analysis for measuring the similarity of document. It is a metric to find similarity between two documents regardless of their size and it is measured by the angular cosine among two vectors determining the pointing of the vectors in the same direction [45]. A smaller angle shows the higher cosine similarity value. This is used for the comparison of two documents. For example, if *X* and *Y* are two vectors representing the documents, then cosine similarity can be found using the following equation.

(8) $$\begin{array}{c} \cos\left(x,y\right)=\frac{X•Y}{\left\|X\right\|\left\|Y\right\|}. \end{array}$$

Here, in the above equation, “•” represents the dot product of the two vectors and “||” shows the length of the vector. Cosine similarity helps identify which users can provide the answers to the question. Or in other words, it can determine the candidate experts for a question to be recommended to the user. In Figure 2, cosine similarity is explained in more detail. As we can see from Figure 2, clustering model will give us the predicted clusters, which may have the same topics as the question. These clusters are mapped with the users' profiles and all the users mapped with predicted clusters are identified as the candidate experts. But these cannot be the right recommendations. These candidate experts are all those users related to clusters identified like clusters *C* and *B*. But not all the users mapped with clusters *C* and *B* can have the same topics as in the question. So, here comes the cosine similarity function, which helps us to identify similar users according to the topics of posted questions from the list of candidate experts.

The article "Combining Latent Factor Model for Dynamic Recommendations in Community Question Answering Forums" was retracted in 2023. Reasons: signs of a paper mill; compromised peer review; unreliable results or conclusions.

For recommendations of the best expertise in a certain topic related to the posted question, three key parameters, reputation of the user, score of the user, and accepted number of answers are used, which can guarantee the best experts recommended to the user which can satisfy the questioner with quality answers. High-level diagram of the proposed approach is shown in Figure 4.

## 4. Results and Discussion

### 4.1. Dataset

To validate and test the proposed methodology, a benchmark dataset is required. In this paper, the dataset from Stack Overflow is used. We have extracted a dataset of 50,000 posts and 20,000 users from Stackexchange archive. This dataset information [46] contains posts and users. A description of data attributes for each user is shown in Table 2.

The dataset is extracted and processed by the methodology to build the user latent profiles, and these profiles are further processed by the recommendation engine to generate recommendations. This latent user profile participates in the recommendation process in two different roles. When a question is fed to the recommendation engine, it analyses the question and finds a similar user having latent trajectories. These similar users are then ranked based on the features, such as reputation, profile score, and number of accepted answers, to make recommendation experience better for the end-user.

The article "Combining Latent Factor Model for Dynamic Recommendations in Community Question Answering Forums" was retracted in 2023. Reasons: signs of a paper mill; compromised peer review; unreliable results or conclusions.

### 4.2. Evaluation Matrices

Evaluation metrics for our system are discussed in detail in this section compared with the baseline approach [31]. The authors have proposed an algorithm named as QRec for finding the potential answerers to the question. The proposed scheme is evaluated by measuring the MRR of the rankings. It is the average of the reciprocal ranks for the results found for all the questions. Although MRR provides the appropriate quality measure for finding the possible answerer, this considers only one highly ranked possible answerer. We have evaluated our model on two bases. First, we have evaluated the throughput of our model in comparison with the baseline approach discussed above. Then, we have evaluated our model based on the quality of prediction using Mean Reciprocal Rank (MRR), Discounted Cumulative Gain (DCG), Mean Average Precision (MAP), and Mean Average Recall (MAR).

#### 4.2.1. Mean Reciprocal Rank (MRR)

MRR is the measure to evaluate a system that creates a list of responses that are arranged by the possibility of correctness for some queries. Reciprocal rank for a query *Q* is the multiplicative inverse of the rank of the first accurate answer. In our case, this metric is the multiplicative inverse of the rank of the first expert found for every topic as shown in the following equation.

(9) $$\begin{array}{c} \text{MRR}=\frac{1}{Q}\sum_{i=1}^{Q}\frac{1}{{\text{Rank}}_{i}}. \end{array}$$

#### 4.2.2. Discounted Cumulative Gain (DCG)

DCG is the foremost standard to evaluate the rank order of the rationality of the expert [28]. Every recommendation is associated with a relevance score and cumulative gain is the sum of all the relevance scores in the set of recommendations.

(10) $$\begin{array}{c} {\text{CG}}_{p}=\sum_{i=1}^{n}{\text{relevance}}_{i}. \end{array}$$

Discounted Cumulative Gain (DCG) is calculated by discounting the relevance score by dividing it with log of the corresponding position as shown in the following equation.

(11) $$\begin{array}{c} \text{DCG}=\sum_{i=1}^{n}\frac{{\text{relevance}}_{i}}{\log_{2}\left(i+1\right)}. \end{array}$$

Here, relevance_*i*_ is the expert score at position *i*.

#### 4.2.3. Mean Average Precision (MAP)

Mean average precision is the mean of the average precision values at ranks of relevant documents, where average precision is the metric of ranked precision that focuses on the highest predicted ranked positions. MAP is a popular metric to evaluate the recommendation systems, which provide a ranked list of recommendations. Precision is defined as the measure that helps to determine the fraction of items recommended, which are relevant out of all the recommended items [47, 48]. Precision can be calculated in recommender systems as in the following equation.

(12) $$\begin{array}{c} \text{Precision}=\frac{\text{relevantrecommendations}}{\text{totalrecommendation}}. \end{array}$$

Average precision value for *N* number of recommendations and *M* number of relevant items can be calculated using the following equation:

(13) $$\begin{array}{c} \text{AveragePrecision}=\frac{1}{M}\sum_{i=1}^{n}\left(pk\right). \end{array}$$

Average precision is useful for a single query whereas to evaluate all the recommendations for all the queries *Q*, Mean of Average Precision is calculated using the formula in the below equation:

(14) $$\begin{array}{c} \text{MAP}=\frac{1}{Q}\sum_{j=1}^{Q}\frac{1}{M}\sum_{i=1}^{n}\left(pk\right). \end{array}$$

The article "Combining Latent Factor Model for Dynamic Recommendations in Community Question Answering Forums" was retracted in 2023. Reasons: signs of a paper mill; compromised peer review; unreliable results or conclusions.

#### 4.2.4. Mean Average Recall (MAR)

Recall is used to measure the proportion of relevant recommendations found from all retrieved recommendations. Recall is a measure to identify the completeness of the recommendations generated [48]. Below is the formula to calculate the recall value of the recommendations:

(15) $$\begin{array}{c} \text{Recall}=\frac{\text{relevantrecommendations}}{\text{totalpossiblerelevantrecommendation}}. \end{array}$$

Average recall value for *N* number of recommendations and *M* number of relevant items can be calculated using following equation:

(16) $$\begin{array}{c} \text{AverageRecall}=\frac{1}{M}\sum_{i=1}^{n}r\left(k\right). \end{array}$$

In the above equation, *r*(*k*) is the recall value at *k* number of recommendations. To evaluate all the recommendations for several queries *Q*, Mean of Average Recall is calculated using formula in the below equation:

(17) $$\begin{array}{c} \text{MAR}=\frac{1}{Q}\sum_{j=1}^{Q}\frac{1}{M}\sum_{i=1}^{n}r\left(k\right). \end{array}$$

## 5. Results

The performance of the recommender engine can be quantified as a function of recommendation generation in the specified period. In the research literature, the throughput is defined as the capability of recommender engine to produce several recommendations per second.  Figure 5 displays the overall effectiveness or performance of our proposed model against the baseline approach. We defined the throughput as a function measuring the number of recommendations generated per second by both engines. We generated a recommendation list and observed the elapsed time of both models. The observations were noted by selecting the random samples from our dataset. From Figure 5, it can be noted that by using the means of clustering approach, the overall throughput of the recommendation engine is exponentially greater than the baseline approach. The reason behind this behaviour is that baseline prediction algorithms do not reduce the neighbourhood for each active user that needs recommendations. The clustering approach is efficient to provide a relevant fraction of neighbours that are candidates for recommendations. Moreover, there is also a relation between throughput and cluster size. We can observe from Figure 5 that as the number of clusters increases, the throughput also gets high. However, this rapid increase in the throughput with cluster numbers is not displayed in the baseline approach. This is due to the reason that traditional recommender engines scan through all the neighbours to find the relevant recommendations, so it does not impact the throughput at all. The topical distribution of the documents given to the LDA model is shown in Figure 6.

The article "Combining Latent Factor Model for Dynamic Recommendations in Community Question Answering Forums" was retracted in 2023. Reasons: signs of a paper mill; compromised peer review; unreliable results or conclusions.

For the measurements of MRR and DCG, firstly, we selected 10 random questions for which the recommended list would be evaluated for both the baseline and proposed model. After identifying topics, the relevance of each question in the sample set is calculated against the topics of each expert in recommendation lists. This process is done for Top 5, Top 10, and Top 15 recommendation lists. The relevance function is defined as the cumulative sum of the weights of the topics that intersect in both question query and recommended user as an expert. A sample of relevance values calculated for one question for Top 5, Top 10, and Top 15; recommendation lists are shown in Tables 3–5, respectively.

However, the range of relevance values is [0, 1], where 0 represents the worst relevance value and 1 for the best relevance value. It can be inferred that those intermediate values can be good or bad depending on their distance from the upper and lower bar. After the relevance calculation for each recommendation list on a query, the relevance values feed to the formula in equation (10). Using equation (10), the values for MRR are calculated for each recommendation lists both for the baseline model and the proposed model.

In the case of finding a list of experts against a question, MRR helps to identify the first user who will answer the question for which the list of answerers is recommended. Although MRR is a better way to identify a good-quality measure of finding potential experts, it focuses only on the one highest expert in the ranked list.  Figure 7 shows that MRR value is higher for the proposed model, which means that recommendation list generated for the questions is more relevant than that of the baseline.

However, there is one key finding that as the recommendation list size increases, there has been decreasing behaviour in the value of MRR for both baseline and proposed model. This is because MRR simply evaluates the rank of highest relevant item in overall recommendation list and counts the reciprocal of it. As the size increases, the probability of high relevance item on more low rank also increases. One such exception in the test scenario can simply make the overall value worst. Since it only counts the evaluation of high-relevance items only, we need a more sophisticated way to incorporate the relevant scores of all items generated in the recommendation list with the query. In research literature, this approach is referred to as a gain of the recommendation list.

The article "Combining Latent Factor Model for Dynamic Recommendations in Community Question Answering Forums" was retracted in 2023. Reasons: signs of a paper mill; compromised peer review; unreliable results or conclusions.

To calculate the quality of ranking, quality of the recommendation list generated by the proposed model DCG is calculated. DCG is advantageous in that it considers the graded values of relevance. Relevance of each of the recommendations from the recommended lists generated for every question from the sample set is calculated. Discounted Cumulative Gain (DCG), which is the discounting of the relevance scores, is then calculated for every list against each question.

It is inferred from Figure 8 that DCG values for the proposed model are much better than that of baseline, which means that the recommendation list generated in the proposed model is more relevant with the question provided as compared to that generated by the baseline model. From Figure 8, it can be inferred that the proposed scheme represents the better rank in each recommendation list size as compared to the baseline.

Furthermore, from Figure 8, it is obvious that as DCG aggregates the gain of each item ranked in the recommendation list, the size of the recommendation list will directly impact the value of DCG in such a way that increased size will represent an increased value of DCG. In that sense to make the comparison clearer, the recommendation list size must be same for both approaches. However, when the size of recommendation list is same, the higher value will represent the higher gain of the recommendation list, making it better in sense of rank. In the same sense, we can claim that for each recommendation list that we used, proposed scheme outperformed the baseline approach.

Mean Average Precision (MAP) and Mean Average Recall (MAR) values are calculated using equations (14) and (17), respectively. Relevance scores found for each recommendation are considered as a true positive value to identify the precision and recall values. (MAP) at *K* and (MAR) at *K* are calculated for *k* number of recommendations in the total *N* number of recommendations, which is shown in Figures 9 and 10, respectively. Graph of (MAP) at *K* goes down as the number of recommendations is increased, which means that for top 5 recommendations, the correctness is more than top 10 recommendations and so on. However, the value of the proposed model is higher than that of the baseline model, which shows that predicted recommendations for proposed models are closer to correctness as compared to the baseline approach. MAR value for the proposed model is higher than that of the baseline model, indicating that the recommendation list generated in the proposed model is closer to completeness than the baseline model.

The article "Combining Latent Factor Model for Dynamic Recommendations in Community Question Answering Forums" was retracted in 2023. Reasons: signs of a paper mill; compromised peer review; unreliable results or conclusions.

## 6. Conclusions

Community question answering (CQA) forums, like Stack Overflow, Quora, Yahoo! Answers, and so on, play an important role in solving the problems people face in their daily life routines. People need to find the experts in these forums to provide the solutions according to their issues. Expert recommendations systems are helping people to solve their problems in many ways. However, all the previous research on these systems is based on the static information available to the systems. People need dynamic solutions according to the updated information provided. This proposed model has considered this issue of dynamicity in these forums by providing an expert recommendation that is somehow more compatible than the previous ones and it provides the dynamic recommendation based on the incremental data without consuming extra time required for the retraining of the model again and again. Instead, we have introduced incremental learning in this platform to avoid the retraining of the models. This model has applied the topic modelling algorithm LDA to extract value topics from the posts extracted from the Stack Overflow website and generate users' profiles by applying the *k*-means clustering approach. We have utilized the features of the Stack Overflow (i.e., the reputation of the user, score, and accepted number of answers for providing the ranked recommendation engine). This model is evaluated based on throughput, MRR, DCG, MAP, and MAR evaluation metrics. The results showed that the proposed model is efficient and promising and provides more quality recommendations than the baseline approach. The overall findings of this research are that incremental clustering introduced in this work is beneficial to efficiency improvisation of the dynamic recommendation systems and this research explores new gaps for the researchers in the field of incremental clustering so that more improvements of the work could be done in a better way.

## 7. Limitations and Future Work

The overall goal of this research was to identify the effect of incremental clustering on the quality of recommendations. Evaluation results of the proposed model against state-of-the-art mechanisms in CQA forums depicted improved quality of recommended experts and an efficient dynamic recommender system. Incremental clustering in the proposed model is applied to the dynamic data and provides efficient results without retraining the model; however, it lacks in different ways. It is done assuming the ideal situation when new coming data points do not affect the scalability of the cluster size and this research does not consider the issues caused due to increasing cluster size. There are many works done for incremental clustering techniques to maintain the scalability and dynamicity issue in the clustering. They can be applied in this research to improve the incremental clustering and overcome its lacks.

The article "Combining Latent Factor Model for Dynamic Recommendations in Community Question Answering Forums" was retracted in 2023. Reasons: signs of a paper mill; compromised peer review; unreliable results or conclusions.

One other issue in this research is the lack of necessary data available at the required time. For example, when a new user joins the community platform who may be an expert in specific field and can provide better answers to the users' questions, the profile of that user will not have much information in it. This will lead to cold start problem where the recommendation system will not recommend him as an expert till the system has extracted the necessary features required for the expert recommendation. This leads to the cold-start problem of the recommendation. There must be some mechanism to deal with such problems of real-time scenarios. A new research direction can be on this issue and research can work on a system able to identify the expertise of the new users adding in the forums. The major focus of the research is to introduce the clustering scheme and verify the usefulness of the clustering in the CQA sites; for this, we applied the traditional *k*-means clustering algorithm. In future research, state-of-the-art techniques of clustering can be applied in CQA sites. Researchers can make some techniques or schemes to determine whether the new user with less information or necessary data available can be recommended as an expert or not. Future research can be done on the techniques to deal with the less information for identification of the expertise.

## Figures and Tables

**Figure 1:** A Typical representation of the recommendation process with user implicit or explicit feedback. User profiles are mapped with user preferences such as interests, history, and attributes.

**Figure 2:** A typical representation of users' latent profile modelling with user implicit or explicit data. User profiles are mapped with user preferences, such as interests, history, and attributes.

**Figure 3:** Elbow method determining the numbers of clusters. An “elbow” effect at value ranges from 35 to 40. The elbow effect indicates that underlying model fits good at a *K*-value of 38.

The article "Combining Latent Factor Model for Dynamic Recommendations in Community Question Answering Forums" was retracted in 2023. Reasons: signs of a paper mill; compromised peer review; unreliable results or conclusions.

**Figure 4:** A pictorial representation of the recommendation engine as a whole system. The recommendation ranking is being based on user feature value.

**Figure 5:** Throughput comparison of the proposed methodology with baseline. The proposed system shows a high number of recommendations generated with an increased number of clusters.

**Figure 6:** Frequency distribution of the user latent profiles for number of documents each user has in the data.

**Figure 7:** Mean reciprocal rank score comparison of the proposed methodology with baseline where user recommendation size = 5, 10, and 15.

**Figure 8:** Discounted cumulative gain score comparison of the proposed methodology with baseline where user recommendation size = 5, 10, and 15.

**Figure 9:** Mean average precision score comparison of the proposed methodology with baseline where user recommendation size = 5, 10, and 15.

**Figure 10:** Mean average recall score comparison of the proposed methodology with baseline where user recommendation size = 5, 10, and 15.

**Algorithm 1:** Latent Dirichlet Allocation.

**Algorithm 2:** Profile segmentation analysis.

**Algorithm 3:** Incremental learning.

**Table 1:** Some typical community question answering forums.

Forum	Launch year	Domain	Language

Wiki Answers	2002	Multiple	English
Yahoo! Answers	2006	Multiple	English
Google Answers	2002	Multiple	Many
Quora	2010	Multiple	English
Stack Overflow	2008	Programming	English
Zhihu	2011	Multiple	Chinese
AnswerBag	2003	Multiple	English

**Table 2:** Description header of the Stack Overflow data attributes for users.

Field name	Description	Value

ID	It is the unique ID of post	27371811
PostTypeId	It shows if a post ID is a question or an answer	2
AcceptedAnswerId	ID of the answer accepted for the question	27371849
ParentId	ID of the original post	27370890
Score	Score given to the post	0
ViewCount	Number of views to a post	166

Body	Body of the post	How to make a while loop with propertiesI have been 2 days playing with iterator, toString parse and a lot of other forms here is theformat I want to display. Work perfect

OwnerUserId	ID of the owner of the post	3072865
Title	Title of the post	Cannot upload full data from excel to database using PHP
Tags	Tags of the post	<csharp><arrays><string>
AnswerCount	Number of answers received for a post	4
CommentCount	Number of comments received for a post	3

**Table 3:** Relevance values for sample recommendation list of proposed model where list size = 5.

User ID	Relevance score

0576	0.7
0087	0.7
1224	0.6
0483	0.8
0192	0.7

**Table 4:** Relevance values for sample recommendation list of proposed model where list size = 10.

User ID	Relevance score

0576	0.7
0087	0.7
1224	0.6
0483	0.8
0192	0.7
0140	0.5
0005	0.4
2135	0.5
2295	0.4
0342	0.4

The article "Combining Latent Factor Model for Dynamic Recommendations in Community Question Answering Forums" was retracted in 2023. Reasons: signs of a paper mill; compromised peer review; unreliable results or conclusions.

**Table 5:** Relevance values for sample recommendation list of the proposed model where list size = 15.

User ID	Relevance score

0576	0.7
0087	0.7
1224	0.6
0483	0.8
0192	0.7
0140	0.5
0005	0.4
2135	0.5
2295	0.4
0342	0.4
1230	0.3
0100	0.3
1960	0.2
0220	0.2
0560	0.2

## Data Availability

Dataset used in this paper is provided and publicly available.
